The article "Disruption of microRNA‐214 during general anaesthesia prevents brain injury and maintains mitochondrial fusion by promoting Mfn2 interaction with Pkm2" was retracted in 2023. Reasons: duplicated images; unreliable results or conclusions.

# Disruption of microRNA‐214 during general anaesthesia prevents brain injury and maintains mitochondrial fusion by promoting Mfn2 interaction with Pkm2

**DOI:** 10.1111/jcmm.15222

**Published:** 2020-11-04

**Authors:** Tiejun Liu, Bin Wang, Gai Li, Xiaoliu Dong, Guannan Yu, Qingzeng Qian, Likun Duan, Hongxia Li, Zhao Jia, Jing Bai

**Affiliations:** ^1^ Department of Anesthesiology North China University of Science and Technology Affiliated Hospital Tangshan China; ^2^ Department of Pediatrics North China University of Science and Technology Affiliated Hospital Tangshan China; ^3^ CT Department North China University of Science and Technology Affiliated Hospital Tangshan China; ^4^ Department of Neurology Tangshan People's Hospital Tangshan China

**Keywords:** brain injury, general anaesthesia, microRNA‐214, mitochondrial fusion, Mitofusin 2, pyruvate kinase M2

## Abstract

Duration of surgical general anaesthesia is associated with severe brain injury and neurological deficits. The specific mechanisms underlying post‐general anaesthesia brain injury, however, still remain to be elucidated. Herein, we explore the role of microRNA‐214 (miR‐214) in the occurrence of brain injury after general anaesthesia and its underlying mechanism. Hippocampal tissues and neurons were isolated from rats exposed to 2% sevoflurane. TUNEL stains reflect hippocampal neuron apoptosis. Cultured hippocampal neurons stained with JC‐1 and MitoTracker dyes were imaged by fluorescence microscope to visualize changes of mitochondrial membrane potential and mitochondrial fusion. Mitochondrial function was evaluated. Mitofusin 2 (Mfn2) binding to miR‐214 or pyruvate kinase M2 (Pkm2) was confirmed by co‐immunoprecipitation, immunofluorescence, dual luciferase reporter gene and RNA immunoprecipitation assays. After exposure to 2% sevoflurane, up‐regulated miR‐214 expression and impaired interaction between Mfn2 and Pkm2 were found in rat hippocampal tissues. Rats exposed to 2% sevoflurane also experienced neuronal injury, mitochondrial defects and deficits in the brain‐derived neurotrophic factor (Bdnf) signalling. miR‐214 was shown to target Mfn2 by impairing its binding with Pkm2. Inhibiting miR‐214 expression using its specific inhibitor improved mitochondrial membrane potential, enhanced mitochondrial fusion, maintained mitochondrial function, restored interaction between Mfn2 and Pkm2, and activated the Bdnf signalling in cultured hippocampal neurons. Adenovirus infection of miR‐214 inhibitor reduced neuron apoptosis and maintained mitochondrial function in the hippocampus of rats exposed to 2% sevoflurane. Taken together, the study demonstrates inhibition of miR‐214 is cerebral protective against brain injury following general anaesthesia.

The article "Disruption of microRNA‐214 during general anaesthesia prevents brain injury and maintains mitochondrial fusion by promoting Mfn2 interaction with Pkm2" was retracted in 2023. Reasons: duplicated images; unreliable results or conclusions.

## 1 INTRODUCTION

Brain injury plagues a large number of patients, which causes both physical and emotional suffering to the patients and their relatives.^1^ It has been reported that patients with brain injury are afflicted by cognitive impairments including deficits in attention and concentration.^2^ The abnormal regulation of mitochondrial dynamic network due to alteration of fusion and fission balance is also responsible for the development of brain injury.^3^ Some of the treatment options being used for brain injury include growth factor therapy as well as the use of mesenchymal stem cells.^4^, ^5^ In addition, the non‐invasive photobiomodulation therapy has been discovered in recent years and becomes possible to establish a novel therapeutic treatment method for brain injury.^6^ Moreover, it is noteworthy that microRNAs (miRs) are involved in the aetiopathology of brain disorders.^7^ Based on the accumulated evidence, it is a promising way to explore the possible regulatory role of miRs in the process of brain injury.

miR‐214 has been identified as a miR that is dysregulated in a variety of pathological conditions and is accountable for the pathogenesis of diverse human disorders.^8^ It has been found that inhibition of miR‐214 expression can alleviate abnormality during neuronal differentiation in neuronal culture models.^9^ Moreover, a previous study has found that up‐regulation of miR‐214 expression is observed in rat models of transient middle cerebral artery occlusion.^10^ Mitofusin 2 (Mfn2) is a type of protein that has been implicated in the process of mitochondrial fusion and associated with alteration in mitochondrial energy supply.^11^ As a member of GTPases, Mfn2 plays an important regulatory role in the fusion machinery of nervous system.^12^ The inhibition of miR‐214 and its interaction with Mfn2 can also serve as a potential target for intervening the pathogenesis of Huntington's disease.^13^ These reports suggested that miR‐214 and Mfn2 may play a contributory role in the pathogenesis of brain diseases. Pyruvate kinase M2 (Pkm2) is a limiting glycolytic enzyme capable of catalysing the last step in glycolysis.^14^ Interestingly, Pkm2 has been found to increase neurogenesis and promote functional recovery in rats after ischaemic stroke.^15^ In addition, Pkm2 can interact with Mfn2 to accelerate mitochondrial fusion, thus, to modulate cancer cell growth.^16^ Herein, the current study was conducted to explore whether miR‐214 could regulate mitochondrial fusion in brain injury *via* regulating Mfn2‐Pkm2 interaction in rats.

## 2 MATERIALS AND METHODS

### 2.1 Animals

Sixty Sprague Dawley (SD) rats (weighing 200‐220 g) of specific‐pathogen‐free grade were purchased from the Laboratory Animal Center of Central South University. Twelve rats were fed in normal air, and the remaining 48 rats were given general anaesthesia (fed in 2% sevoflurane for 90 minutes). Adenovirus vectors were injected into rats every 3 days after sevoflurane anaesthesia. On the 7th day after anaesthesia, all rats were killed after bloodletting *via* the eyeballs. Brain tissues were then isolated, part of which were fixed in 10% neutral formalin solution for 24 hours, dehydrated using gradient alcohol and cleared with xylene. Then, these tissues were embedded in a paraffin tank and sliced into paraffin blocks, which were then cryopreserved in liquid nitrogen for further use. The current study conformed to the guidelines approved by North China University of Science and Technology Affiliated Hospital. All animal experiments were conducted according to the international conventions on laboratory animal ethics and relevant national regulations. All efforts were made to minimize the suffering of the included animals.

The article "Disruption of microRNA‐214 during general anaesthesia prevents brain injury and maintains mitochondrial fusion by promoting Mfn2 interaction with Pkm2" was retracted in 2023. Reasons: duplicated images; unreliable results or conclusions.

### 2.2 Construction of adenovirus vectors

AdP14ARF (Shanghai Genechem Co., Ltd.) was chosen for the recombinant adenovirus vector construction labelled by green fluorescent protein. AdP14ARF vectors containing miR‐214 inhibitor or negative control (NC) inhibitor were injected into the brain of rats exposed to 90‐minutes 2% sevoflurane.

### 2.3 Cell treatment

After disinfection using 75% ethanol, the whole brains of 1‐day‐old SD rats were isolated by detaching scalp and skull. With the blunt separation of hippocampus and removal of blood vessels, the hippocampus was cut into blocks (diameter = 0.4 mm) and reacted with 0.25% (g/L) trypsin and 0.04 (g/L) DNAase for 12 minutes. The detachment was terminated by horse serum. The tissue blocks were treated to disperse cells. The cell suspension was added in minimum Eagle's medium (MEM) containing 10% foetal bovine serum (FBS), 5% horse serum, 25 mmol/L KCl, 10 mmol/L 2‐[4‐(2‐hydroxyethyl)piperazin‐1‐yl]ethanesulphonic acid, 105 U/L penicillin and 0.1 g/L streptomycin. After filtering through a 75‐µm nylon mesh, the cell suspension was incubated on a 35‐mm petri dish coated with poly‐L‐lysine in an incubator at 37°C with 5% CO_2_ and 95% O_2_ under saturated humidity at a density of 0.6 × 10^9^ cells/L. On the 3rd day, 5 µmol/L cytarabine was supplemented for further 24‐hours incubation. The medium was then renewed with Dulbecco's Modified Eagle Medium (DMEM) containing 10% FBS and penicillin/streptomycin. The hippocampal neurons on the 7th day after culture were identified by neuron‐specific enolase immunocytochemical staining using streptavidin‐peroxidase.

The article "Disruption of microRNA‐214 during general anaesthesia prevents brain injury and maintains mitochondrial fusion by promoting Mfn2 interaction with Pkm2" was retracted in 2023. Reasons: duplicated images; unreliable results or conclusions.

The Mfn2 and Pkm2 overexpression plasmids were purchased from GenePharma Co., Ltd.. Neurons were inoculated into 6‐well plates with a cell density of 3 × 10^5^ neurons/well. When the cell confluence reached about 50% ‐ 60%, Lipofectamine 2000 kit (Invitrogen) was used for transfection.

### 2.4 Haematoxylin‐eosin (HE) staining

Hippocampal tissues were collected and sliced into 4 µm sections. The sections were stained with haematoxylin solution for 3 minutes and eosin solution for 5 minutes. Finally, the sections were observed under an optical microscope (XP‐330, Shanghai Bingyu Optical Instruments Co., Ltd.).

### 2.5 Enzyme‐linked immunosorbent assay (ELISA)

The eyeballs of the rat were allowed to rest overnight at 4°C. The following day, the eyeballs were centrifuged at 3500 × *g* to extract the clear upper‐layer serum. The levels of interleukin‐6 (IL‐6) and tumour necrosis factor‐α (TNF‐α) in the cell lysate of both normal rats and rats exposed to 2% sevoflurane were then detected using IL‐6 and TNF‐α ELISA kits MSKbio. Cell culture medium was collected after 24 hours of cell incubation, followed by centrifugation at 1000 × *g* at room temperature for 10 minutes. The supernatant was extracted and used to determine the levels of TNF‐α and IL‐6. Finally, the standard curve was drawn in strict accordance with the procedures provided on the ELISA kit instructions.

### 2.6 Measurement of mitochondrial oxidative respiratory activity

The oxidative respiratory activity of brain mitochondria was measured by oxygen electrode method. A total of 0.7 mL of reaction medium was added to the reaction pool (total volume: 0.8 mL; temperature: 28°C) and incubated under air‐saturated conditions for 2 minutes. Next, 0.1 mL of mitochondrial suspension (containing 0.1 mg mitochondrial protein) was added to the pool, followed by the addition of 10 µL oxidized substrates (0.5 mol/L sodium malate and 0.5 mol/L sodium pyruvate) with 1‐minutes incubation, and another addition of 5 µL of 0.1 mol/L adenosine diphosphate. The oxygen consumption curve was recorded and calculated based on the respiratory rate after addition of adenosine diphosphate (referred to as ST3) as well as after adenosine diphosphate depletion (referred to as ST4). ST3 and ST4 were expressed by the mole number [nmol/O min.mg protein] of oxygen atoms consumed by per milligram of mitochondrial protein per unit time, and the ratio between ST3 and ST (ST3/ST4) was indicative of mitochondrial respiratory control rate.

### 2.7 Terminal deoxynucleotidyl transferase‐mediated 2'‐deoxyuridine 5'‐triphosphate nick end labelling (TUNEL) staining

The paraffin sections were dewaxed and hydrated in the same way as mentioned above. Following rinsing with 3% hydrogen peroxide for 10‐15 minutes, 20 µg/mL of protease K that had been dissolved in Tris/HCl was added to the sections for incubation at room temperature for 15‐30 minutes. Next, TUNEL reaction mixture was added to the sections for incubation in a wet box at 37°C for 60 minutes. Finally, the sections were observed under a fluorescence microscope.

The article "Disruption of microRNA‐214 during general anaesthesia prevents brain injury and maintains mitochondrial fusion by promoting Mfn2 interaction with Pkm2" was retracted in 2023. Reasons: duplicated images; unreliable results or conclusions.

### 2.8 Measurement of mitochondrial superoxide dismutase (SOD) activity and reduced glutathione (GSH) and malondialdehyde (MDA) content

The substantia nigra (125 mm^3^ in size) was taken from the hippocampus of rats with different treatment. A total of 1 mL phosphate buffer saline (PBS) homogenate was added to the substantial nigra, followed by centrifugation at 12 000 × *g* at 42°C for 10 minutes. Following extraction of the supernatant, the protein concentration was measured using a bicinchoninic acid detection kit (P0011, Beyotime) and the content of MDA (A003‐1‐2), SOD (A001‐3‐2) and GSH (A006‐2‐1) in the hippocampus was determined using the MDA, SOD and GSH kit (Nanjing Jiancheng Bioengineering Institute.

Neurons were inoculated into 6‐well culture plates at a cell density of 6 × 10^4^ cells/mL. The contents of SOD, MDA and GSH were measured according to kits’ instructions (Nanjing Jiancheng Bioengineering Institute).

### 2.9 JC‐1 staining

Neurons were inoculated into 6‐well culture plates at a cell density of 6 × 10^4^ cells/mL. Then, 2 mL of culture medium was added into each well. The neurons were then added with JC‐1 at a final concentration of 1 µg/mL at 37°C and washed twice with 1 × PBS. Following incubation for 30 minutes, mitochondrial fluorescence intensity (at excitation wavelength of 488 nm; at emission wavelength of 595 nm and 525 nm) was measured under a fluorescence microscope (ECLIPSE Ti, Nikon).

### 2.10 Counting of mitochondria

Neurons were inoculated into 6‐well culture plates at a cell density of 6 × 10^4^ cells/mL. Then, 2 mL of culture medium was added into each well. After rinsed twice with 1 × PBS, MitoTracker at a final concentration of 1 µg/mL was added to the neurons at 37°C and incubated for 0.5 hour. Finally, the mitochondria were observed under a Nikon‐Ti fluorescence microscope.

### 2.11 Co‐immunoprecipitation (Co‐IP)

The rat brain tissues were cut into pieces and then placed in a centrifugal tube containing radioimmunoprecipitation assay solution. The homogenate was prepared at 4°C, followed by centrifugation at 14 000 × *g* for 10 minutes. Following the removal of the precipitates, the extracted supernatant was added into a 1.5 mL centrifugal tube containing 1 µL specific antibody, followed by addition of pre‐treated 50 µL protein A/G agarose beads. Next, the precipitated complex was extracted and subject to subsequent Western blot analysis relative to immunoglobulin G (IgG).

The article "Disruption of microRNA‐214 during general anaesthesia prevents brain injury and maintains mitochondrial fusion by promoting Mfn2 interaction with Pkm2" was retracted in 2023. Reasons: duplicated images; unreliable results or conclusions.

### 2.12 Dual luciferase reporter gene assay

The wild‐type (WT) and mutant‐type (MUT) reporter plasmids of Mfn2 (WT‐Mfn2 and MUT‐Mfn2) were designed and supplied by GenePharma. The NC mimic and miR‐214 mimic were cotransfected with WT‐Mfn2 and MUT‐Mfn2 into rat hippocampal neurons, respectively. After being cultured for 48 hours, the neurons were collected and the luciferase activity was detected by dual luciferase reporter gene assay according to the manufacturer's instructions provided by GeneCopoeia's dual luciferase detection kit (D0010, Solarbio). Meanwhile, the 20/20 Luminometer (E5311, Zhongmei Biotechnology Co., Ltd.) was employed to detect the luminescence signal.

### 2.13 RNA immunoprecipitation (RIP) assay

The binding of miR‐214 and Mfn2 was detected using a RIP kit (Millipore Corp of Billerica). Neurons were lysed using an equal amount of radioimmunoprecipitation assay lysis (P0013B, Beyotime Biotechnology Co.) on an ice bath for 5 minutes, followed by centrifugation at 16 000*g* for 10 minutes to collect the supernatant. Part of the cell extract was taken out and used as input, while the other part was co‐precipitated with antibody and magnetic beads for incubation. The magnetic bead‐antibody complex was rinsed and re‐suspended in 900 µL RIP Wash Buffer. The samples were placed on magnetic pedestals in order to collect the bead‐protein complex. The precipitated complex and input were treated with protease K; then, RNA was subsequently extracted to determine the expression of miR‐214 and Mfn2 by quantitative polymerase chain reaction (qPCR) detection. The antibodies used in RIP were rabbit anti‐Argonaute2 (Ago2, 1 µL/mL, ab3238, Abcam Inc, Cambridge, UK), and rabbit anti‐IgG (ab109489; dilution ratio of 1:100, Abcam) was used as NC.

### 2.14 Immunohistochemistry

The paraffin‐embedded sections of normal rats and rats exposed to 2% sevoflurane were routinely dewaxed and hydrated. The sections were dewaxed with xylene I and II for 10 minutes each, treated with gradient alcohol (100%, 95%, 80% and 70%; 2 minutes each) and immersed in 3% hydrogen peroxide for 10 minutes. Next, high‐pressure antigen retrieval was conducted for 90 seconds, and the sections were then cooled at room temperature and sectioned following a rinse with PBS. Afterwards, 5% bovine serum albumin solution was added to the sections for incubation at 37°C for 30 minutes, followed by further incubation with 50 mL rabbit antimouse polyclonal antibodies against Mfn2 (5 µg/mL, ab56889, Abcam) and Pkm2 (5 µg/mL, ab206130, Abcam) at 4°C overnight. Subsequently, 50 µL biotinylated rat anti‐goat antibody to IgG (RXE0155, dilution ratio of 1:100, Rongchuang Biotechnology Co., Ltd.) was added to the sections for incubation at 37°C for 30 minutes. The sections were colourized with diaminobenzidine, counterstained using haematoxylin for 5 minutes, rinsed using tap water, dehydrated, cleared, sealed and examined under an optical microscope (XP‐330, Shanghai Bingyu Optical Instrument Co., Ltd.). PBS was used as the primary antibody in replacement of NC. A positive percentage of more than 10% among the neurons was indicative of positive expression, where the staining was mainly in the cytoplasm or cell membrane, presenting in brown‐yellowish colouration. The positive expression rates of Mfn2 and Pkm2 were observed in 5 high‐power randomly chosen microscopic fields.

The article "Disruption of microRNA‐214 during general anaesthesia prevents brain injury and maintains mitochondrial fusion by promoting Mfn2 interaction with Pkm2" was retracted in 2023. Reasons: duplicated images; unreliable results or conclusions.

### 2.15 Immunofluorescence

Rat brain sections were dewaxed and detached using complex enzymes at room temperature for 1 minutes and washed with PBS for 3 minutes. The sections were then immersed in 0.01 mol/L sodium citrate repair solution, subjected to microwave retrieval at a medium‐high temperature for 30 minutes, rewarmed for 30‐60 minutes and permeabilized with 0.3% Triton × 100 at room temperature for 20 minutes. Afterwards, normal goat serum was used to seal the sections for 20 minutes, followed by incubation with primary antibodies to Mfn2 (5 µg/mL, ab56889, Abcam) and Pkm2 (5 µg/ml, ab85555, Abcam) at 4°C overnight. After incubation, the fluorescent secondary antibody was added to the sections and further incubated at 37°C for 1 hour. After staining using 4',6‐diamidino‐2‐phenylindole for 30 minutes, anti‐fade mounting medium was used to seal the sections, and the sections were lastly observed under a Nikon‐Ti fluorescence microscope.

### 2.16 Reverse transcription qPCR (RT‐qPCR)

The total RNA was extracted from the cultured neurons using the Trizol kit. The primer sequences (Table 1) for miR‐214 and Mfn2 were designed by Takara. The obtained RNA was reversely transcribed into complementary DNA (cDNA) according to the manufacturer's instructions of the PrimeScript RT reagent kit (RR036A, Takara). Subsequently, real‐time fluorescence qPCR was performed using a SYBR^®^ Premix Ex TaqTM II kit (RR820A, Takara) on a fluorescence qPCR device. Finally, the relative expression of miR‐214 and Mfn2 was calculated using the 2^−ΔΔ^ *^C^* ^t^ method with U6 and β‐actin serving as the internal reference.

**Table 1:** Primer sequences for RT‐qPCR

Target	Forward primer (5′‐3′)	Reverse primer (5′‐3′)
miR‐214	GCGGCACAGCAGGCACAGACA	CCAGTGCAGGGTCCGAGGTA
Mfn2	ATGATAGACGGCTTGAA	CGACTCCCTCTTTGTGA
U6	CTCGCTTCGGCAGCACA	AACGCTTCACGAATTTGCGT
β‐actin	AGGGAAATCGTGCGTGACAT	GAACCGCTCATTGCCGATAG

Note

RT‐qPCR, reverse transcription‐quantitative polymerase chain reaction.

The article "Disruption of microRNA‐214 during general anaesthesia prevents brain injury and maintains mitochondrial fusion by promoting Mfn2 interaction with Pkm2" was retracted in 2023. Reasons: duplicated images; unreliable results or conclusions.

Abbreviations: MFN2, Mitofusin 2; miR, microRNA.

### 2.17 Western blot analysis

Cells were lysed with radioimmunoprecipitation lysis (R0010, Solarbio) containing phenylmethylsulphonyl fluoride. A total of 50 µg proteins were subjected to sodium dodecyl sulphate‐polyacrylamide gel electrophoresis. Next, the proteins were wet‐transferred onto a nitrocellulose membrane and then incubated with the primary antibodies, including rat anti‐human antibodies to Mfn2 (1 µg/mL, ab56889), Pkm2 (1 µg/mL, ab206130), brain‐derived neurotrophic factor (Bdnf; ab108319, dilution ratio of 1:1000), cAMP response element‐binding protein (Creb; ab178322, dilution ratio of 1:500), phosphorylated‐Cerb (p‐Cerb; ab32096, dilution ratio of 1:1000) and glyceraldehyde‐3‐phosphate dehydrogenase (GAPDH; ab9485, dilution ratio of 1:1000) at 4°C overnight. All aforementioned antibodies were purchased from Abcam Inc. The membrane was rinsed thrice with Tris‐Buffered Saline Tween‐20 (each time 5 minutes) and incubated with horseradish peroxidase‐labelled goat anti‐rabbit secondary antibody to IgG (HA1003, dilution ratio of 1:100, Yanhui Biotechnology) at room temperature for 1 hour. Subsequently, the membrane was developed using an enhanced chemiluminescence reagent (ECL808‐25, Biomiga) for 1 minutes, covered with a plastic film and exposed to X‐ray film (36209ES01, Shanghai Qcbio Science & Technologies co. Ltd.). With GAPDH used as the internal reference, the ratio of grey value between target band and internal reference band was reported as the relative protein expression.

### 2.18 Statistical analysis

Statistical analyses were conducted using the SPSS 22.0 software (IBM Corp.). All measurement data were presented as mean ± standard deviation. The data between two groups obeying normal distribution and homogeneous variance in unpaired design were compared using unpaired *t* test. Comparisons among multiple groups were assessed by one‐way analysis of variance (ANOVA). Tukey's was employed for post hoc test. A value of *P* < .05 was considered as statistically significant.

## 3 RESULTS

### 3.1 miR‐214 was overexpressed in rat hippocampus after general anaesthesia accompanied by brain injury

The expression of miR‐214 in normal rats and rats exposed to 2% sevoflurane was determined by RT‐qPCR with the result found that the expression of miR‐214 in the rats exposed to 2% sevoflurane significantly increased when compared to the normal rats (*P* < .05) (Figure 1A). HE staining was used to detect brain tissue injury in rats. The neurons in normal rats were arranged neatly, the nuclei were clear and the cytoplasm was uniformly stained. In contrast, the brain tissues of the rats exposed to 2% sevoflurane showed loose neuronal arrangement in different degrees, swelling and degeneration of neurons, nuclear pyknosis and hyperchromatism of cytoplasm (Figure 1B). The levels of IL‐6 and TNF‐α in peripheral blood of both normal rats and rats exposed to 2% sevoflurane were detected by ELISA with the results clarified that the levels of IL‐6 and TNF‐α in the rats exposed to 2% sevoflurane were significantly higher than those in normal rats (*P* < .05) (Figure 1C). In addition, neuronal apoptosis was observed using TUNEL staining. Results showed that TUNEL apoptotic‐positive neurons in rats exposed to 2% sevoflurane were significantly higher than those in normal rats (*P* < .05) (Figure 1D). In comparison with that of the normal rats, the content of SOD and GSH in rats exposed to 2% sevoflurane was significantly lower, while the level of MDA was significantly higher (*P* < .05). The results of mitochondrial oxidative respiratory activity presented that when compared with the normal rats, the rats exposed to 2% sevoflurane exhibited significantly lower mitochondrial respiratory control ratio, along with significantly inhibited mitochondrial oxidative respiratory activity (*P* < .05) (Figure 1F). Meanwhile, the protein expression of Bdnf and Creb was detected by Western blot analysis. Results revealed that relative to the normal rats, the rats exposed to 2% sevoflurane exhibited a significant decrease in the protein expression of Bdnf and Creb (*P* < .05), as well as in the extent of Creb phosphorylation (*P* < .05) (Figure 1G).

The article "Disruption of microRNA‐214 during general anaesthesia prevents brain injury and maintains mitochondrial fusion by promoting Mfn2 interaction with Pkm2" was retracted in 2023. Reasons: duplicated images; unreliable results or conclusions.

**Figure 1:** Overexpression of miR‐214 and brain injury are observed in hippocampus of rats after general anaesthesia. A, The expression of miR‐214 in brain tissues of normal rats and rats exposed to 2% sevoflurane determined by RT‐qPCR. B, The rat brain tissue injury in normal rats and rats exposed to 2% sevoflurane detected by HE staining (× 200). C, The expression of pro‐inflammatory cytokines (IL‐6 and TNF‐α) in the peripheral blood of normal rats and rats exposed to 2% sevoflurane determined by ELISA. D, Measurement of neuronal apoptosis in normal and rats exposed to 2% sevoflurane detected by TUNEL assay (×400). E, The contents of SOD, GSH and MDA in brain tissues of normal rats and rats exposed to 2% sevoflurane. F, Mitochondrial oxidative respiratory activity in brain tissues of normal rats and rats exposed to 2% sevoflurane. G, The protein expression of Bdnf and Creb, as well as the extent of Creb phosphorylation normalized to GAPDH in brain tissues of normal rats and rats exposed to 2% sevoflurane determined by Western blot analysis. *P < .05 vs normal rats. The data were measurement data and expressed as mean ± standard deviation. The data between two groups obeying normal distribution and homogeneous variance in unpaired design were compared using unpaired *t* test (n = 12)

The article "Disruption of microRNA‐214 during general anaesthesia prevents brain injury and maintains mitochondrial fusion by promoting Mfn2 interaction with Pkm2" was retracted in 2023. Reasons: duplicated images; unreliable results or conclusions.

### 3.2 General anaesthesia impaired Mfn2 interaction with Pkm2 in rats

Subsequently, the expression of Mfn2 and Pkm2 in normal rats and rats exposed to 2% sevoflurane was detected by immunohistochemistry and Western blot analysis. Compared with the normal rats, the rats exposed to 2% sevoflurane showed significant decrease in the expression of Mfn2 and Pkm2 (Figure 2A and B). In addition, the results of Co‐IP revealed that the enrichment of Pkm2 protein in pull‐down samples using Mfn2 antibody was significantly lower when compared to IgG (*P* < .05) (Figure 2C). Moreover, the localization of Mfn2 and Pkm2 was detected using a fluorescent double‐labelling technique. Based on the results (Figure 2D), the co‐localization fluorescence intensity was significantly weaker in the rats exposed to 2% sevoflurane when compared to the normal rats (*P* < .05). The above results indicated that general anaesthesia affected the interaction between Mfn2 and Pkm2.

**Figure 2:** General anaesthesia impairs Mfn2 interaction with Pkm2 in rats. A, The expression of Mfn2 and Pkm2 in normal rats and rats exposed to 2% sevoflurane detected by immunohistochemistry (×400). *P < .05 vs the normal rats. B, The expression of Mfn2 and Pkm2 normalized to GAPDH in normal rats and rats exposed to 2% sevoflurane determined by Western blot analysis. *P < .05 vs the normal rats. C, The interaction between Mfn2 and Pkm2 verified by Co‐IP. *P < .05 vs IgG. D, The co‐localization of Mfn2 and Pkm2 detected using fluorescent double‐labelling technique (×400). *P < .05 vs the normal rats. The data were measurement data and expressed as mean ± standard deviation. The data between two groups obeying normal distribution and homogeneous variance in unpaired design were compared using unpaired *t* test (n = 12)

### 3.3 miR‐214 negatively modulated Mfn2 expression

Dual luciferase reporter gene assay was performed to detect the targeting relationship between miR‐214 and Mfn2 (Figure 3A). Results showed that cotransfection of miR‐214 mimic and Mfn2‐WT resulted in a significant decrease in the luciferase activity of Mfn2‐WT (*P* < .05), but no significant change was detected in luciferase activity of Mfn2‐MUT during cotransfection of miR‐214 mimic and Mfn2‐MUT. Moreover, RIP assay showed more miR‐214 immuno‐coprecipitating with Mfn2 relative to IgG (*P* < .05) (Figure 3B). Furthermore, the expression of Mfn2 was detected by RT‐qPCR and Western blot analysis with the result displayed that the expression of Mfn2 was significantly up‐regulated by miR‐214 inhibitor (*P* < .05) (Figure 3C and D). Overall, it was concluded that miR‐214 could target Mfn2 and inhibit its expression.

The article "Disruption of microRNA‐214 during general anaesthesia prevents brain injury and maintains mitochondrial fusion by promoting Mfn2 interaction with Pkm2" was retracted in 2023. Reasons: duplicated images; unreliable results or conclusions.

**Figure 3:** miR‐214 negatively modulates Mfn2 expression. A, The targeting relationship between miR‐214 and Mfn2 predicted by dual luciferase reporter gene assay. *P < .05 vs NC mimic. B, The binding sites between miR‐214 and Mfn2 verified by RIP. *P < .05 vs IgG. C, The expression of Mfn2 determined by RT‐qPCR. *P < .05 vs NC inhibitor. D, The protein expression of Mfn2 normalized to GAPDH determined by Western blot analysis. *P < .05 vs NC inhibitor. The data were measurement data and expressed as mean ± standard deviation. The data between two groups obeying normal distribution and homogeneous variance in unpaired design were compared using unpaired *t* test. The cell experiment was repeated three times independently

### 3.4 Disturbing miR‐214 maintained mitochondrial fusion *via* Mfn2‐Pkm2 interaction

The rat primary neurons were isolated and cultured. The identification of rat hippocampal neurons showed that the neuron‐specific enolase reaction products were presented with brown colour, evenly distributed in the cytoplasm, accompanied by protuberances, and the nucleus was stained in blue. The cultured neurons were identified as the positive neurons (Figure 4A). Subsequently, overexpression or silencing of miR‐214/Mfn2/Pkm2 was transfected into the neurons. ELISA (Figure 4B) was performed to determine the levels of cytokines (IL‐6 and TNF‐α) in neurons in response to different treatments, followed by the measurement of MDA, SOD and GSH levels in transfected neurons (Figure 4C). Based on the results, the delivery of miR‐214 mimic contributes to marked elevation in the levels of IL‐6 and TNF‐α (*P* < .05), as well as the MDA content (*P* < .05), accompanied by a decline in SOD and GSH content (*P* < .05). By contrast, the overexpression of Mfn2 caused a notable decrease in the levels of IL‐6 and TNF‐α (*P* < .05), and MDA content (*P* < .05), as well as an increase in SOD and GSH content (*P* < .05). Moreover, the delivery of miR‐214 inhibitor led to a significant decrease in the levels of IL‐6 and TNF‐α (*P* < .05), reduced MDA content (*P* < .05) and elevated SOD and GSH content (*P* < .05), while silencing of Pkm2 showed an opposite trend (*P* < .05). Furthermore, the combination of miR‐214 mimic and Mfn2 overexpression have resulted in significantly lower levels of IL‐6 and TNF‐α (*P* < .05), lower content of MDA (*P* < .05), and higher SOD and GSH content (*P* < .05) when compared to the treatment of miR‐214 mimic alone (*P* < .05). Besides, in comparison with treatment of miR‐214 inhibitor alone, the combination of miR‐214 inhibitor and Mfn2 silencing has resulted in significantly higher levels of IL‐6 and TNF‐α, higher content of MDA (*P* < .05), and lower SOD and GSH content (*P* < .05). Subsequently, the mitochondrial membrane potential changes were assessed using JC‐1 staining (Figure 4D) and MitoTracker staining (Figure 4E), and the mitochondrial fusion was observed under a laser confocal microscope. Results showed that the highest mitochondrial membrane potential was detected in normal rats (detected as red fluorescence), accompanied by normal mitochondrial fission. Rat neurons treated with miR‐214 inhibitor or Mfn2 expressing plasmid showed the second highest mitochondrial membrane potential, accompanied by normal mitochondrial fission. However, 2% sevoflurane‐induced rat neurons treated with miR‐214 mimic and Mfn2 expressing plasmid or treated with miR‐214 mimic and Pkm2 expressing plasmid showed a relatively lower mitochondrial membrane potential, along with inhibited mitochondrial fission compared with normal rat neurons. The lowest mitochondrial membrane potential was found in rat neurons with miR‐214 mimic or silenced Pkm2, accompanied by significant inhibition of mitochondrial fission. Furthermore, the protein expression of Pkm2, Mfn2, Bdnf and Cerb along with the extent of Cerb phosphorylation was determined using Western blot analysis (Figure 4F). Results revealed that the protein expression of Pkm2, Mfn2, Bdnf and Cerb as well as the extent of Cerb phosphorylation was significantly decreased by miR‐214 mimic (*P* < .05) but increased by Mfn2 overexpression (*P* < .05). Moreover, addition of miR‐214 inhibitor resulted in an increase in the protein expression of Pkm2, Mfn2, Bdnf and Cerb as well as elevated extent of Cerb phosphorylation (*P* < .05), which could be notably reversed by the silencing of Pkm2 (*P* < .05). The combined treatment of miR‐214 mimic and Mfn2 overexpression led to the elevated protein expression of Pkm2, Mfn2, Bdnf and Cerb accompanied by increased extent of Cerb phosphorylation (*P* < .05) relative to treatment of miR‐214 mimic alone (*P* < .05). Besides, when compared to the treatment of miR‐214 inhibitor alone, the delivery of both miR‐214 inhibitor and silenced Mfn2 contributed to reduced protein expression of Pkm2, Mfn2, Bdnf and Cerb along with diminished extent of Cerb phosphorylation (*P* < .05). After silencing of miR‐214, Co‐IP assay was performed to detect the binding of Mfn2 with Pkm2, with the results found that treatment of miR‐214 inhibitor led to the decreased binding of Mfn2 with Pkm2, suggesting that miR‐214 could block the interaction between Mfn2 and Pkm2 (Figure 4G). The above results demonstrated that mitochondrial fusion could be suppressed by miR‐214 through Mfn2‐Pkm2 interaction.

The article "Disruption of microRNA‐214 during general anaesthesia prevents brain injury and maintains mitochondrial fusion by promoting Mfn2 interaction with Pkm2" was retracted in 2023. Reasons: duplicated images; unreliable results or conclusions.

**Figure 4:** Disturbing miR‐214 maintains mitochondrial fusion via Mfn2‐Pkm2 interaction. A, The identification results of rat hippocampal neurons. B, The expression of pro‐inflammatory cytokines (IL‐6 and TNF‐α) in rat neurons in response to different treatments determined by ELISA. C, The contents of MDA, SOD and GSH in rat neurons in response to different treatments. D, Mitochondrial membrane potential changes in rat neurons in response to different treatments assessed by JC‐1 staining. E, Mitochondrial fusion in rat neurons in response to different treatments detected by MitoTracker staining (×400). F, The protein expression of Pkm2 and Mfn2 normalized to GAPDH in rat neurons in response to different treatments determined by Western blot analysis. G, The interaction between Mfn2 and PKM2 with miR‐214 inhibitor detected by Co‐IP. * *P* < .05 vs NC mimic + oe‐NC. #*P* < .05 vs NC inhibitor + si‐NC. &*P* < .05 vs miR‐214 mimic + oe‐NC. @*P* < .05 vs miR‐214 inhibitor + si‐NC. The data were measurement data and expressed as mean ± standard deviation. The data among multiple groups were analysed by ANOVA. Tukey's was utilized for post hoc test. The cell experiment was repeated three times independently

### 3.5 Disturbing miR‐214 ameliorated brain injury in rats following general anaesthesia

The expression of miR‐214 was determined by RT‐qPCR. Results showed that the expression of miR‐214 was significantly diminished after treatment with miR‐214 inhibitor (*P* < .05) (Figure 5A). Subsequently, immunohistochemistry was employed to determine the expression of Mfn2 (Figure 5B). Results revealed that the positive expression of Mfn2 was up‐regulated in response to miR‐214 inhibitor (*P* < .05). Moreover, the levels of IL‐6 and TNF‐α in peripheral blood of rats in response to different treatments were detected by ELISA (Figure 5C). Besides, the levels of IL‐6 and TNF‐α significantly decreased in the presence of miR‐214 inhibitor (*P* < .05). TUNEL staining showed that apoptosis of neurons treated with miR‐214 inhibitor significantly reduced (*P* < .05) (Figure 5D). The delivery of miR‐214 inhibitor also contributed significantly to the elevation of SOD and GSH content, as well as reduction in MDA content (Figure 5E). Furthermore, the protein expression of Bdnf, and Creb, as well as the extent of Cerb phosphorylation was determined using Western blot analysis. Results showed that the protein expression of Bdnf, Creb and the extent of Creb phosphorylation increased with the presence of miR‐214 inhibitor (*P* < .05) (Figure 5F). The above results collectively demonstrated that low expression of miR‐214 could alleviate brain injury in anaesthetized rats.

The article "Disruption of microRNA‐214 during general anaesthesia prevents brain injury and maintains mitochondrial fusion by promoting Mfn2 interaction with Pkm2" was retracted in 2023. Reasons: duplicated images; unreliable results or conclusions.

**Figure 5:** Adenovirus infection of miR‐214 inhibitor ameliorates brain injury in rats following general anaesthesia. A, The expression of miR‐214 in brain tissues of rats undergoing different treatments determined by RT‐qPCR. B, The expression of Mfn2 in brain tissues of rats undergoing different treatments detected by immunohistochemistry (×400). C, The expression of pro‐inflammatory cytokines (IL‐6 and TNF‐α) in the peripheral blood of rats undergoing different treatments determined by ELISA. D, Measurement of neuronal apoptosis in rats undergoing different treatments detected by TUNEL assay (×400). E, The content of SOD, GSH and MDA in brain tissues of rats undergoing different treatments. F, The protein expression of Bdnf, Creb and the extent of Creb phosphorylation normalized to GPADH in brain tissues of rats undergoing different treatments determined by Western blot analysis. *P < .05 vs NC inhibitor. The data were measurement data and expressed as mean ± standard deviation. The data between two groups obeying normal distribution and homogeneous variance in unpaired design were compared using unpaired *t* test (n = 12)

## 4 DISCUSSION

Emerging evidence suggests that miRNAs may play a potential role in brain injury.^17^ Herein, this study aimed to explore the effect of miR‐214 on the pathogenesis of brain injury. Our results demonstrated that down‐regulated miR‐214 could activate Mfn2‐Pkm2 interaction by up‐regulating the expression of Pkm2 and thereby facilitate mitochondrial fusion and further alleviate brain injury after general anaesthesia.

Interestingly, this study found that miR‐214 was highly expressed while Mfn2 was poorly expressed in rat models after general anaesthesia. Accumulated experiments have demonstrated that general anaesthetics usually cause detrimental effects on the brain especially following administration to infants or elderly adults.^18^ It has been reported that anaesthesia can affect mRNA expression after traumatic brain injury in mice.^19^ The up‐regulation of miR‐214 has been found in many diseases. For instance, miR‐214 is highly expressed in the sera of elderly patients with acute myocardial infarction.^20^ Moreover, the up‐regulation of miR‐214‐3p is also observed in the medial prefrontal cortex of chronic social defeat stress rats, while inhibition of miR‐214‐3p can reverse the resultant depressive‐like behaviours,^21^ which is consistent with our results. Furthermore, findings from another study are also in line with our results, where the decline in Mfn2 expression is found at the stage of reperfusion, while the overexpressed Mfn2 can confer mitochondrial protection to the reperfusion‐mediated cerebral injury.^22^ Additionally, the protein level of Mfn2 shows a reduction in fibroblast production from patients with sporadic Alzheimer's disease.^23^

The article "Disruption of microRNA‐214 during general anaesthesia prevents brain injury and maintains mitochondrial fusion by promoting Mfn2 interaction with Pkm2" was retracted in 2023. Reasons: duplicated images; unreliable results or conclusions.

Another important finding was that the interaction between Mfn2 and Pkm2 after general anaesthesia was discovered using Co‐IP and fluorescent double‐labelling technique. Moreover, results from dual luciferase reporter gene assay showed that miR‐214 could target Mfn2, which was further verified by RIP assay. In addition, the results from RT‐qPCR and Western blot analysis also demonstrated that miR‐214 could down‐regulate the expression of Mfn2. Furthermore, our results demonstrated that the inhibition of miR‐214 could reverse mitochondrial fusion. Similar to our result, the increased level of Mfn2 induced by LIG *via* promotion of mitochondrial fusion and reduction of mitochondrial fission is observed and may be responsible for dynamics of mitochondrial morphology.^24^ In consistent with our result, the overexpressed Pkm2 has been reported to be capable of facilitating mitochondrial fusion by weakening p53 stability.^25^ The down‐regulated Pkm2 protein has been found in the hippocampus of neonatal brain injury post‐anaesthesia induced by ketamine in animals.^26^ Moreover, both protein and mRNA levels of Pkm2 are down‐regulated in the occurrence of middle cerebral artery occlusion.^27^ Available evidence has indicated that miR‐214 down‐regulates Pkm2 in non‐small‐cell lung cancer cells.^28^ Besides, it has been reported that overexpressed Pkm2 can up‐regulate Mfn2 expression via miR‐106b to be implicated in the mediation of mitochondrial fusion.^29^ In the current study, it was found that the down‐regulated miR‐214 was able to activate Mfn2‐Pkm2 interaction by increasing the expression of Pkm2 as well as contributed to the up‐regulation of mitochondria fusion protein Mfn2 expression, thereby facilitating mitochondria fusion.

In addition, the down‐regulated miR‐214 was found to ameliorate brain injury, which was reflected by improved mitochondrial function, reduced pro‐inflammatory cytokines (IL‐6 and TNF‐α), increased in the content of SOD and GSH and decreased in the content of MDA, along with increased protein expression of Bdnf, Creb and the extent of Creb phosphorylation. It was concluded that the regulatory role of Mfn2‐Pkm2 interaction in brain injury was resulted from the activation of Mfn2‐Pkm2 interaction that inhibited miR‐214 expression. Previous studies have discovered the similar role of Mfn2 and Pkm2 in the regulation of mitochondria dysfunction. For instance, instead of neuron protection, Mfn2 is capable of protecting dopaminergic neurons in idiopathic Parkinson's disease.^30^ Besides, early treatment of Pkm2 can provide acute neuroprotection against ischaemic brain damage, and the delayed treatment brings about a better functional recovery in the post‐stroke brain.^15^ Similarly, the reduced expression of Pkm2 in the mitochondria treated with shikonin has been reported to aggravate the oxidative stress and nutrient deficiency, thereby promoting mitochondria dysfunction in hepatocellular carcinoma.^31^ In addition, the presence of the reduced fusion protein Mfn2 in post‐cardiac arrest is observed along with an increasing number of fragmented mitochondria.^32^ Consistently, the increased expression of miR‐214 in Huntington's disease cell models results in altered mitochondrial morphology and deregulated cell cycle by targeting Mfn2.^13^ These previous reports may support our findings that the down‐regulation of miR‐214 may contribute to the beneficial effects in brain injury protection *via* Mfn2‐Pkm2 interaction.

The article "Disruption of microRNA‐214 during general anaesthesia prevents brain injury and maintains mitochondrial fusion by promoting Mfn2 interaction with Pkm2" was retracted in 2023. Reasons: duplicated images; unreliable results or conclusions.

## 5 CONCLUSIONS

To conclude, the down‐regulated miR‐214 could ameliorate brain injury after general anaesthesia by promoting Mfn2‐Pkm2 interaction *via* up‐regulation of Pkm2 expression, which contributed to the promotion of mitochondrial fusion (Figure 6). These results indicate that the regulatory role of miR‐214 may well serve as a potential therapeutic strategy for protection against brain injury.

**Figure 6:** The mechanism of miR‐214 in the regulation of brain injury with the involvement of Mfn2/Pkm2 interaction. General anaesthesia promotes the expression of miR‐214, while the down‐regulation of miR‐214 up‐regulates the Mfn2 expression to promote the interaction between Pkm2 and Mfn2, thereby facilitating the mitochondrial fusion in rats following general anaesthesia

## CONFLICT OF INTEREST

None.

## AUTHOR CONTRIBUTIONS

Tiejun Liu, Qingzeng Qian and Likun Duan designed the study. Tiejun Liu, Bin Wang and Gai Li collated the data, carried out data analyses and produced the initial draft of the manuscript. Xiaoliu Dong, Guannan Yu, Hongxia Li and Zhao Jia contributed to drafting the manuscript. Jing Bai revised the figures and table. All authors have read and approved the final submitted manuscript.

## Data Availability

Research data not shared.

## References

[1] Bharadwaj VN , Nguyen DT , Kodibagkar VD , Stabenfeldt SE . Nanoparticle‐Based Therapeutics for Brain Injury. Adv Healthc Mater. 2017;7:1700668.10.1002/adhm.201700668PMC590367729034608

The article "Disruption of microRNA‐214 during general anaesthesia prevents brain injury and maintains mitochondrial fusion by promoting Mfn2 interaction with Pkm2" was retracted in 2023. Reasons: duplicated images; unreliable results or conclusions.

[2] Gocheva V , Hund‐Georgiadis M , Hediger K . Effects of animal‐assisted therapy on concentration and attention span in patients with acquired brain injury: a randomized controlled trial. Neuropsychology. 2018;32:54‐64.2903506810.1037/neu0000398

[3] Fan LF , He PY , Peng YC , et al. Mdivi‐1 ameliorates early brain injury after subarachnoid hemorrhage via the suppression of inflammation‐related blood‐brain barrier disruption and endoplasmic reticulum stress‐based apoptosis. Free Radic Biol Med. 2017;112:336‐349.2879001210.1016/j.freeradbiomed.2017.08.003

[4] Larpthaveesarp A , Ferriero DM , Gonzalez FF . Growth factors for the treatment of ischemic brain injury (growth factor treatment). Brain Sci. 2015;5:165‐177.2594268810.3390/brainsci5020165PMC4493462

[5] Hasan A , Deeb G , Rahal R , et al. Mesenchymal stem cells in the treatment of traumatic brain injury. Front Neurol. 2017;8:28.2826525510.3389/fneur.2017.00028PMC5316525

[6] Wang R , Dong Y , Lu Y , et al. Photobiomodulation for global cerebral ischemia: targeting mitochondrial dynamics and functions. Mol Neurobiol. 2019;56:1852‐1869.2995194210.1007/s12035-018-1191-9PMC6310117

[7] Kuss AW , Chen W . MicroRNAs in brain function and disease. Curr Neurol Neurosci Rep. 2008;8:190‐197.1854111410.1007/s11910-008-0031-0

[8] Zhao Y , Ponnusamy M , Zhang L , et al. The role of miR‐214 in cardiovascular diseases. Eur J Pharmacol. 2017;816:138‐145.2884212510.1016/j.ejphar.2017.08.009

[9] Mellios N , Feldman DA , Sheridan SD , et al. MeCP2‐regulated miRNAs control early human neurogenesis through differential effects on ERK and AKT signaling. Mol Psychiatry. 2018;23:1051‐1065.2843910210.1038/mp.2017.86PMC5815944

[10] Herzog R , Zendedel A , Lammerding L , Beyer C , Slowik A . Impact of 17beta‐estradiol and progesterone on inflammatory and apoptotic microRNA expression after ischemia in a rat model. J Steroid Biochem Mol Biol. 2017;167:126‐134.2788472710.1016/j.jsbmb.2016.11.018

[11] Yu HY , Guo YH , Gao W . [Mitochondrial fusion protein Mfn2 and cardiovascular diseases]. Sheng Li Ke Xue Jin Zhan. 2010;41:11‐16.21417008

[12] Jahani‐Asl A , Cheung EC , Neuspiel M , et al. Mitofusin 2 protects cerebellar granule neurons against injury‐induced cell death. J Biol Chem. 2007;282:23788‐23798.1753772210.1074/jbc.M703812200

[13] Bucha S , Mukhopadhyay D , Bhattacharyya NP . Regulation of mitochondrial morphology and cell cycle by microRNA‐214 targeting Mitofusin2. Biochem Biophys Res Commun. 2015;465:797‐802.2630753610.1016/j.bbrc.2015.08.090

[14] Dong G , Mao Q , Xia W , et al. PKM2 and cancer: the function of PKM2 beyond glycolysis. Oncol Lett. 2016;11:1980‐1986.2699811010.3892/ol.2016.4168PMC4774429

The article "Disruption of microRNA‐214 during general anaesthesia prevents brain injury and maintains mitochondrial fusion by promoting Mfn2 interaction with Pkm2" was retracted in 2023. Reasons: duplicated images; unreliable results or conclusions.

[15] Chen D , Wei L , Liu ZR , et al. Pyruvate Kinase M2 Increases Angiogenesis, Neurogenesis, and Functional Recovery Mediated by Upregulation of STAT3 and Focal Adhesion Kinase Activities After Ischemic Stroke in Adult Mice. Neurotherapeutics. 2018;15:770‐784.2986905510.1007/s13311-018-0635-2PMC6095793

[16] Li T , Han J , Jia L , et al. PKM2 coordinates glycolysis with mitochondrial fusion and oxidative phosphorylation. Protein Cell. 2019;10:583‐594.3088744410.1007/s13238-019-0618-zPMC6626593

[17] Atif H , Hicks SD . A Review of MicroRNA Biomarkers in Traumatic Brain Injury. J Exp Neurosci. 2019;13:1179069519832286.3088652510.1177/1179069519832286PMC6410383

[18] Vutskits L . General anesthetics in brain injury: friends or foes? Curr Pharm Des. 2014;20:4203‐4210.24025058

[19] Staib‐Lasarzik I , Kriege O , Timaru‐Kast R , et al. Anesthesia for euthanasia influences mRNA expression in healthy mice and after traumatic brain injury. J Neurotrauma. 2014;31:1664‐1671.2494508210.1089/neu.2013.3243PMC4170812

[20] Yin Y , Lv L , Wang W . Expression of miRNA‐214 in the sera of elderly patients with acute myocardial infarction and its effect on cardiomyocyte apoptosis. Exp Ther Med. 2019;17:4657‐4662.3108659710.3892/etm.2019.7464PMC6489010

[21] Deng ZF , Zheng HL , Chen JG , et al. miR‐214‐3p targets beta‐catenin to regulate depressive‐like behaviors induced by chronic social defeat stress in mice. Cereb Cortex. 2019;29:1509‐1519.2952217710.1093/cercor/bhy047

[22] Lan S , Liu J , Luo X , Bi C . Effects of melatonin on acute brain reperfusion stress: role of Hippo signaling pathway and MFN2‐related mitochondrial protection. Cell Stress Chaperones. 2019;24:235‐245.3063206410.1007/s12192-018-00960-2PMC6363627

[23] Martin‐Maestro P , Gargini R , Garcia E , et al. Slower dynamics and aged mitochondria in sporadic Alzheimer's disease. Oxid Med Cell Longev. 2017;2017:9302761.2920127410.1155/2017/9302761PMC5672147

[24] Xu YJ , Mei Y , Qu ZL , et al. Ligustilide ameliorates memory deficiency in APP/PS1 transgenic mice via restoring mitochondrial dysfunction. Biomed Res Int. 2018;2018:4606752.3007934710.1155/2018/4606752PMC6069587

[25] Wu H , Yang P , Hu W , et al. Overexpression of PKM2 promotes mitochondrial fusion through attenuated p53 stability. Oncotarget. 2016;7:78069‐78082.2780166610.18632/oncotarget.12942PMC5363644

[26] Zhao CH , Li GH , Wang Q , Zhao B , Wang ZB . Mechanisms of propofol attenuation of ketamine‐induced neonatal brain injury. Eur Rev Med Pharmacol Sci. 2016;20:133‐137.26813465

[27] Zeng X , Liu N , Zhang J , et al. Inhibition of miR‐143 during ischemia cerebral injury protects neurones through recovery of the hexokinase 2‐mediated glucose uptake. Biosci Rep. 2017;37:BSR20170216.2852255110.1042/BSR20170216PMC6434090

The article "Disruption of microRNA‐214 during general anaesthesia prevents brain injury and maintains mitochondrial fusion by promoting Mfn2 interaction with Pkm2" was retracted in 2023. Reasons: duplicated images; unreliable results or conclusions.

[28] Zhang K , Zhang M , Jiang H , et al. Down‐regulation of miR‐214 inhibits proliferation and glycolysis in non‐small‐cell lung cancer cells via down‐regulating the expression of hexokinase 2 and pyruvate kinase isozyme M2. Biomed Pharmacother. 2018;105:545‐552.2988637510.1016/j.biopha.2018.06.009

[29] Wu H , Li Z , Wang Y , et al. MiR‐106b‐mediated Mfn2 suppression is critical for PKM2 induced mitochondrial fusion. Am J Cancer Res. 2016;6:2221‐2234.27822413PMC5088287

[30] Zhao F , Wang W , Wang C , et al. Mfn2 protects dopaminergic neurons exposed to paraquat both in vitro and in vivo: implications for idiopathic Parkinson's disease. Biochim Biophys Acta Mol Basis Dis. 2017;1863:1359‐1370.2821557810.1016/j.bbadis.2017.02.016PMC5474135

[31] Yang J , Cong X , Ren M , et al. Circular RNA hsa_circRNA_0007334 is predicted to promote MMP7 and COL1A1 expression by functioning as a miRNA sponge in pancreatic ductal adenocarcinoma. J Oncol. 2019;2019:7630894.3142815110.1155/2019/7630894PMC6681607

[32] Li Y , Tang Q , Wang P , et al. Dynamic changes of mitochondrial fusion and fission in brain injury after cardiac arrest in rats. Biomed Res Int. 2017;2017:1948070.2944573210.1155/2017/1948070PMC5763114

